The article "Multidrug-Resistant Biofilm, Quorum Sensing, Quorum Quenching, and Antibacterial Activities of Indole Derivatives as Potential Eradication Approaches" was published in 2022. Journal: Biomed Res Int.

# Multidrug-Resistant Biofilm, Quorum Sensing, Quorum Quenching, and Antibacterial Activities of Indole Derivatives as Potential Eradication Approaches

**DOI:** 10.1155/2022/9048245

**Published:** 2022-08-24

**Authors:** Ayodele T. Odularu, Anthony J. Afolayan, Alexander P. Sadimenko, Peter A. Ajibade, Johannes Z. Mbese

**Affiliations:** ^1^Department of Chemistry, Faculty of Science and Agriculture, University of Fort Hare, Private Bag X1314, Alice 5700, South Africa; ^2^School of Further and Continuing Education, Faculty of Science and Agriculture, University of Fort Hare, Private Bag X1314, Alice 5700, South Africa; ^3^Centre of Phytomedicine, Department of Botany, Faculty of Science and Agriculture, University of Fort Hare, Alice 5700, Private Bag X1314, South Africa; ^4^School of Chemistry and Physics, University of KwaZulu-Natal, Pietermaritzburg Campus, Scottsville 3209, South Africa

## Abstract

Challenges encountered in relapse of illness caused by resistance of microorganisms to antimicrobial agents (drugs) are due to factors of severe stress initiated by random use of antibiotics and insufficient beneficial approaches. These challenges have resulted to multiple drug resistance (MDR) and, subsequently, biofilm formation. A type of intercellular communication signal called quorum sensing (QS) has been studied to cause the spread of resistance, thereby enabling a formation of stable community for microorganisms. The QS could be inhibited using QS inhibitors (QSIs) called quorum-quenching (QQ). The QQ is an antibiofilm agent. Indole derivatives from plant sources can serve as quorum-quenching eradication approach for biofilm, as well as a promising nontoxic antibiofilm agent. In other words, phytochemicals in plants help to control and prevent biofilm formation. It could be recommended that combination strategies of these indoles' derivatives with antibiotics would yield enhanced results.

## 1. Introduction

Microorganisms' resistance to multidrugs is a global public health challenge [1–4]. These microorganisms (bacteria, fungi, parasites, viruses, and nonpharmaceuticals) have corresponding antimicrobial agents (antibacterial, antifungal, antiparasitic, and nonpharmaceutical agents) [4, 5].

According to Singh et al., the sphere's archaea and bacteria exclusively comprise prokaryotic microorganisms, while algae, fungi, protozoa, slime molds, and water moulds are eukaryotic microbes [6]. Archaea and bacteria represent the majority of life forms on our planet. Recently, an estimation anticipated 1011–1012 microbial species on Earth with 99.9% microbial species yet to be laboratory cultured [6]. Additionally, the existing antimicrobial agents reduced in their effectiveness, and some of these microorganisms were virtually untreatable because of the challenge of increase in pathogens resistance [7–10]. This challenge might be due to factors, such as demanding stress initiated by unselective use of antibiotics and insufficient beneficial approaches [11, 12].

Bacteria, being the most populated among these microorganisms commensurate with their highest biofilm formation [6]. Proffering reasonable solution to eradicating this highest biofilm formation has resulted to the focus in this research. One of the reasons of their highest population was as a result of failure to treat bacterial infections, such as nosocomial infections warranting them to form biofilms [13–24]. Nosocomial infections are also called hospital acquired infections or healthcare-associated infections (HAI or HCAI). The study is aimed at assessing biofilm formation in context and quorum sensing (QS), relationship between biofilm and antibiotic resistance pattern, biofilm formation's mechanism of action, several biofilms' eradication approaches, and the distinct contributions of indole' derivatives as stakeholders to eradicating biofilm.

## 2. Biofilm Formation in Context and Quorum Sensing (QS)

### 2.1. Biofilm Formation in Context

Almost all bacterial species composed of pathogens have the ability to form biofilms [25]. Bacterial biofilms introduce a big health challenge because of their very high resistances to many types of therapeutics, including conventional antibiotics [25]. In 1674, Antonie Van Leuwenhoek used his primitive microscopic to observe biofilms [26], although Bill Costerton coined the term, “biofilm” in 1978 [27].

According to Chen and Wen's perspective, bacterial biofilm is a particular kind of persistent bacterial infection [16]. Berlanga and Guerrero stated that biofilms are heterogeneous structures consisting of diverse microorganism populations encircled by a matrix (typical of exopolysaccharides), which permits their attachments to inert (for example, glass, plastic, and rocks) or organic (for example, cuticle, mucosa, and s kin) surfaces [27]. Biofilm is defined as an assemblage of microbial cells which is irreversibly surface associated and matrix walled with polysaccharide materials [28]. Wolska et al. defined biofilms as structured ecosystems where microbes attach to surfaces and entrench in a matrix consisting eDNA, polysaccharides, and proteins, as well as their growths on a multistep process [25].

Microbes could attach to both nonliving and living surfaces, such as indwelling medical devices, industrial and potable water system piping, natural aquatic systems, living tissues, and prosthetics to form a biofilm consisting of extracellular polysaccharides, proteins, and other constituents [16, 26, 28–31]. On development matter, biofilm development is in stages and some factors control the formation [26]. Berlanga and Guerrero specified that biofilm development is in three unique stages of attachment, maturation (active sessile cells), and release [27]. However, Tilahun et al. and Wolska et al. stated that biofilm developed in five stages (reversible attachment, irreversible attachment, maturation I, maturation II, and dispersion) [25, 26]. Four factors, which significantly contribute and control biofilm formation, are genetics (bacterial motility, cell membrane proteins, extracellular polysaccharides, and signaling molecules) and environment (nutrients, oxygen, pH, and temperature) [25, 26].

Biofilm-associated organisms are quite different from their freely suspended counterparts referred to as planktonic bacteria, with respect to their transcribed genes [28]. In terms of growth types, bacteria switch between two growth types, namely, the unicellular life phase, where bacterial cells are free-swimming (planktonic), and multicellular life phase, where bacterial cells are sessile and live in a biofilm [27]. In the switching cycle, bacteria complete two biological alterations through gene communication: (i) from planktonic cells to sessile cells inside a biofilm and (ii) from sessile to isolated, new planktonic cells [27].

#### 2.1.1. Community Signaling Agents

Community signaling agents are referred to as quorum sensing (QS). Quorum sensing (QS) is a process where bacteria communicate with one another using community signaling agents.

*(1) Quorum Sensing*. Seven groups of researchers gave similar definitions to quorum sensing. Monte et al. defined QS as a mechanism by which a bacterial population observes its cell division [32]. The mechanism controls bacterial biofilm development and growth. It is also related to cell-cell interactions, which depends on some factors, such as synthesis, exchange, and awareness of small signal molecules between bacteria [32]. Solano et al., in line with Monte et al.'s definition for QS, defined QS as a cell-cell interaction mechanism that synchronizes gene expression in response to population cell density [33]. Jung et al. defined QS as a microbial signaling communication approach for monitoring complexity and population density among bacterial cells [34]. Kemp et al. defined QS as a type of intercellular communication numerous bacterial species used to produce and secrete signaling molecules to influence development and growth in a bacterial population [35]. Chen and Wen defined QS as a microbial cell-to-cell communication system selected for cell-density and/or population-based gene regulation [16]. Gupta et al. defined QS as a community accord among microorganisms and referred to it as chemical signaling among microorganisms [36]. Pena et al. defined quorum sensing (QS) as a communication mechanism between bacteria that allows certain processes, such as biofilm formation, virulence factor manifestation, secondary metabolites' production, and stress alteration mechanisms, such as bacterial competition mechanisms entailing secretion systems (SS) [37].

As soon as there is an accumulated signal threshold, specific virulence characters are controlled in bacteria in response to the immediate environment [36]. These virulence characters are recognized to contribute to pathogenic bacteria diseases [36]. The SSs are everywhere and are found in both Gram-negative and Gram-positive bacteria [37, 38]. They have an essential role in bacterial communication and worldwide roles which contribute to pathogenesis and virulence [37]. The communication among bacterial cells through QS depends on autoinducers [34, 39]. These autoinducers are the production, secretion, and detection of small molecules [34, 39]. Jung et al. stated that a minimum of four parallel signaling pathways come together to control a single regulator activity to modify its QS response in the human pathogen called Vibrio cholera [34].

Based on types of QS systems, some main types of QS systems recognized and characterized are N-acyl-homoserine lactone (AHL) systems (Gram negative bacteria), 4-quinolone systems (Gram negative bacteria, hydrophobic signal), AgrD peptide systems (Gram positive bacteria), and Al2/LuxS systems (both Gram negative bacteria and Gram-positive bacteria). The AHL quorum-sensing mutant lasl formation of a thin biofilm was more sensitive to treatment by antibiotics and sterilization solutions [16, 40, 41]. The introduction of a functional lasl or addition of a suitable AHL could complement the phenotype [16]. On the other hand, Gram-positive bacteria use autoinducing peptides (AIP) as their autoinducers [42, 43]. Once Gram-positive bacteria detect high concentrated AIP in the environment, AIP binds to a receptor to trigger kinase [42–47]. The kinase introduces a phosphate group as a transcription factor, which controls gene transcription, also called a two-component system [48, 49]. The additional promising mechanism is the AIP transport to the cytosol, which binds directly to a transcription factor to start or inhibit transcription [42, 50].

Based on applications of QS, Chen and Wen stated that the application of QS system helps individual cells to make and discharge signal and identify the signal in the neighboring environment simultaneously [16]. Additionally, quorum sensing (QS) was used to regulate the biofilm maturation phase [16]. However, Wolska et al. stated that quorum sensing, cyclic guanosine-5′-monophosphate, and small RNAs are the main regulators to biofilm formation [25].

Concisely, this Section 2.1. gives Bill Corsterson as the name inventor for biofilm, Antonie Van Leuwenhoek, as the observer of biofilm with a microscope, four definitions of biofilm (gritty bacterial infections including nosocomial infections made up of polysaccharide), biofilm formation on nonliving and living surfaces, biofilm's three or five stages of development controlled by four genetic and four environmental factors, biofilm's transcription genes, biofilm's growth rate, biofilm constituents, and biofilm effects on hosts. In Section 2.1.1., all the seven groups of researchers regarded QS as signaling communication mechanisms among bacteria in biofilm formation. Additionally, the QS has different types as regards bacterial strain and applied to regulate biofilm maturation via development and growth stages.

### 2.2. Relationship between Biofilm and Antibiotic Resistance Pattern

This biofilm formation might stimulate drug resistance and inflammation causing persistent infections in their hosts [16, 51, 52]. Based on enhanced and increased antibacterial drug resistance, recently, there was an increase in biofilm formation by a class of clinically relevant bacteria referred to as ESKAPE (Enterococcus faecalis, Staphylococcus aureus, Klebsiella pneumoniae, Acinetobacter baumannii, Pseudomonas aeruginosa, and Enterobacter spp.) resulting in high mortality [29, 30, 53, 54].

The expansion and increase of biofilm with beta-lactamases producing strains both led to the widespread distribution of multidrug-resistant Gram-negative bacilli. Gram-negative bacilli are the general causative agents for community-acquired nosocomial and opportunistic infections [55]. The relationship between biofilm formation and antimicrobial resistance varies with every bacterium species [55]. However, Dumaru et al. stated that no relationship could be observed between multidrug resistance or worldwide resistance and biofilm formation [56]. This study agrees with Cepas et al. that acquirement of a particular antimicrobial resistance could assist or improve biofilm formation in numerous Gram-negative bacteria [55]. However, multidrug-resistant isolates do not exhibit a trend to being greater biofilm producers than non-multiresistant isolates [55]. For instance, Pseudomonas aeruginosa is an opportunistic Gram-negative pathogen known for its acquired and intrinsic antibiotic resistance. It has notorious capability to form biofilm, which usually assists chronic infections [57].

Ahmed et al. observed a higher resistance proportion of antibiotics called ciprofloxacin (CIP) in the CIP-evolved biofilm populations than in planktonic populations exposed to the same drug concentrations. However, the minimum inhibition concentrations (MICs) of ciprofloxacin were lower in CIP-resistant isolates chosen from the planktonic cultures [57]. Ahmed et al. discovered common evolutionary paths between the various lineages, with mutations in identified CIP resistance determinants, growth condition-dependent adaptations, and a loss of virulence-linked traits in the populations that evolved in the absence of antibiotics [57]. They concluded that biofilms could assist in the development of low-level mutational resistance, possibly because of lower efficient drug exposure than in planktonic cultures [57]. Qui et al. assessed the relationship between antibiotic resistance, biofilm formation, and biofilm-specific resistance in clinical 272 isolates of Acinetobacter baumannii sampled from different hospitals in China from 2010 to 2013 [58]. They implied from their study that biofilm acted as a mechanism to enhance bacteria survival in isolates with both not high enough resistance level and very weak high enough resistance level [58]. In summary, there is a specific relationship between biofilm formation and antimicrobial resistance to every Gram-negative bacterium specie, as observed in enhanced and increased antibacterial drug resistance in ESKCAPE. This confirms biofilm relationship with the multidrug resistance of bacteria to antibiotics.

### 2.3. Biofilm Formation's Mechanism of Action

The mechanisms by which antibiotic resistance develops are essential in determining the survival of biofilm microbes. The microbes that form biofilm naturally experience high mutation, which enables them to grow resistant mechanisms providing chance for genes to develop enzymes that deactivates the antibiotics or extrudes the antibiotics by efflux pumps [22]. Among bacterial species, the four main mechanisms developed for antibiotic resistance are (i) altering cell permeability to constrain the antibiotics influx to the cells, (ii) making the antibiotics-bound cellular targets passive by modifying them, (iii) making antibiotics ineffectual with enzymatic cleavage, and (iv) controlling of efflux pumps to oust the antibiotics from the cellular membrane [22].

## 3. Antibiofilm Agents' Division into Different Groups via Mechanism of Action

The QS is often involved in the pathogenesis activation; therefore, inhibition of quorum sensing provides a potential treatment mechanism for bacterial infections. Various ways to inhibit these QS systems are signal molecule synthesis inhibition, signal function impairment, or with signal receptors' interference [35]. Mechanism of action of antibiofilm agent for biofilm inhibition is adhesion inhibitors, cyclic diguanylate inhibitors, efflux pump inhibitors, extracellular polymeric substance synthesis inhibitors, and quorum sensing inhibitor. Emergent biofilm mechanism actions such as small synthetic molecule inhibitors, antimicrobial peptides (AMPs), bioactive compounds isolated from fungi, nonproteinogenic amino acids and antibiotics, efflux pump inhibitors (EPIs), free fatty acids, such as oleic acid and cis-2-decenoic acid, ionic liquids (for instance, 1-alkylquinolinum bromide), nature-derived bioactive scaffolds, natural phytoconstituents (natural compounds isolated from bacteria, marine, and plants), quaternary ammonium compounds (QACs), and quorum-quenching agents are in approval to eradicate the resistance [29, 30, 35]. Natural products are small molecular secondary metabolites, such as alkaloids, flavonoids, and terpenoids required for plants' survival [59, 60]. They are used as therapeutic for human beings.

## 4. Eradication Approaches

Biofilms have negative and positive features in homes and industries [26]. As regards the positive features of biofilm, some of the essential characteristics of biofilm bacteria are of biotechnological importance, such as the synthesis of valued compounds (for example, surfactants and ethanol) and the improvement/processing of specific foods, such as table olives. The ecology of biofilm formation would enable the systems' design which could make interested products and enhance their yields [27]. In line with the aim of this study, the negative features of biofilms are reviewed and their eradication approaches.

### 4.1. Combination Strategies, Targeting Biofilm Phenotype, and Targeting Community Signaling Agents as Eradication Approaches

Sharma and Yadav emphasized that efficient control of biofilm would need a combined effort to develop therapeutic agents to target the biofilm phenotype [31]. In addition, they stated that inhibition of community signaling-based agents is needed to prevent the formation or boost biofilms' detachment [31]. In support of Sharma and Yadav, as well as Tilahun et al. stated that a combination of physical and chemical methods was needed to eliminate biofilm [26, 31].

#### 4.1.1. Combination Strategies

Combination strategies used as ways to eradicate biofilm are (i) mechanical disruption or removal by sonication, (ii) immune modulation (azithromycin (C38H72N2O12) and low-dose doxycycline (C22H24N2O8), (iii) antimicrobial agents (silver (Ag)) and tobramycin (C18H37N5O9), and (iv) amphotericin B lipid formulations and the echinocandins against the Candida biofilms [31]. In support of Sharma and Yadav's study, Beitelshees et al. concluded that a combinational approach should be adopted to offer full shield against biofilm-forming bacteria and their resulting diseases [61]. Rephrasing Beitelshees et al., increasing biofilm surface separation with combination approaches might offer worldwide protection against biofilm forming bacterial diseases [61].

#### 4.1.2. Targeting Biofilm Phenotype

Previously, there was less focus on the relationship between a bacterial phenotype and the organism's pathogenesis [61]. Recently, the research confirmed that biofilm acts as a principal period of pathogenesis for approximately 80% of bacterial diseases [61]. Some biofilms called microbiomes do not lead to direct disease formation but are accountable for disorders in the local environment, such as disease-causing contaminations or automated disturbance to trigger a phenotypic shift [61]. This shift leads to the dispersal of virulent bacteria from the biofilm. The phenotype shift has been in a relationship with the upregulation of virulence factors, which allows the bacteria to spread into usually sterilized areas, such as the blood, brain, lungs, and middle ear, thereby causing clinical conditions entailing bacteremia, bacterial meningitis, pneumonia, and otitis media correspondingly. There are several bacterial species cycles between growth phases and biofilm formation [61].

These phases could be commonly characterized by one or more cellular phenotype(s), each with unique virulence factor functionality [61]. Additionally, several phenotypes could mostly be observed in the phases, which could depend on host conditions or the presence of nutrients and oxygen terrains in the biofilm, that is, the microenvironment [61]. Presently, most antibiofilm approaches have targeted a single phenotype [61]. The approaches have compelled efficient, yet partial protection because of their inadequate consideration of gene expression dynamics throughout the bacteria's pathogenesis [61]. Roy et al. stated that biofilms shield the attacking bacteria against the host's immune system through damaged activation of phagocytes and complement system [62]. In summary, the consideration of various phenotypes detected in biofilms is important to develop efficient therapeutic approaches against biofilm-forming bacteria.

#### 4.1.3. Targeting Community Signaling Agents

*(1) Quorum-Quenching (QQ) and Antibiofilm Agents*. The quorum-sensing inhibition (QSI) is in diverse means via strategic approach, such as quorum quenching (QQ). The QQ is used to avoid the initiation of its virulence factors and has been well thought out as an alternative therapy to avoid the adverse effects of antibiotic overuse [36]. There is a rationale between naturally evolved quorum-quenching strategies and synthetically modified methods approved to eliminate QS and its signaling pathways ([8, 34, 37–41, 62–66]; and [67]). Rahin et al. stated that present research was aimed at developing nontoxic antibiofilm agents to disperse, inhibit, or prevent biofilms [29, 30]. Additionally, the current antibiofilm agents consist of moieties, such as bromopyrrole, furanone, imidazole, indole, peptides (D-amino acids), phenols, sulfide, and triazole., possess the potential to disperse bacterial biofilms in vivo and might absolutely influence human medicine in the future [29, 30].

In summary, eradication approaches to control biofilm are either combination strategies, targeting the biofilm phenotype, targeting community signaling agents to prevent biofilm formation, but the focus of this study was to use targeting community signaling agents with phytochemicals to prevent biofilm formation.

## 5. Phytochemical (Plant Sources) as a Quorum-Quenching Eradication Approach for Biofilm

Present research reveals that compounds of plants origin known as phytochemicals could help to reduce the danger of developing diseases, such as cancer, diabetes mellitus, hypertension, and microorganisms [68–70]. Plants are major sources of efficient antimicrobial products for numerous organisms entailing bacteria, fungi, insects, nematodes, yeasts, and other plants [32]. To discover new antimicrobial agents with innovative action modes, phytochemicals in plants were explored as foundation for the identification of original and active antimicrobials [32, 71, 72]. Phytochemicals are defined as chemicals made by plants to shield themselves from environmental hitches, such as predators [73]. Other researchers confirmed that phytochemicals could be obtained from natural products, such as plants [71, 74].

However, Ajuru et al. stated that, depending on the source, some bioactive compounds are either sourced from animals or plant-based compounds (phytochemicals) [73]. In line with this, phytochemicals, also referred to as photobiotic or phytogenic, are natural bioactive compounds sourced from plants [69]. Phytochemicals can prevent peptidoglycan synthesis, harm microbial membrane structures, transform bacterial membrane surface hydrophobicity, and modify quorum sensing (QS) [32]. To counteract the biofilm resistance challenges, Borges et al. used phytochemicals as novel approaches to eliminating bacterial quorum sensing (QS) signaling pathways and provided ways to inhibit or eliminate biofilm's basic phenotypes [75]. Other approaches are the application of phytochemicals as chelating agents and efflux pump inhibitors [75].

From the opinions of Monte et al., Altemimi et al., and Srivastava et al., and other researchers, this study reviews the intervention of phytochemicals to control and seek a solution to biofilms' eradication [32, 69, 71–73, 75].

### 5.1. Mechanism of Action of Indole Derivatives

According to Lee et al., indole derivatives are prevalent in both prokaryotic and eukaryotic communities. However, there is a very limited knowledge about their mechanisms of action [76].

### 5.2. Intervention of Indole and Its Derivatives

Indole is a group of phytochemicals related to microorganisms' prevention [77–81].

Indole is an aromatic hydrocarbon consisting of a benzene ring fused with a pyrrole ring. Over eighty-five species of Gram-positive and Gram-negative bacteria produce indole with numerous and various functions in bacterial signaling [82]. Apart from its anticancer properties, anti-inflammatory properties, antimicrobial properties, controlling biofilm formation, responses to stress, and virulence the transition from exponential to stationary phase, it also facilitates signaling between enteric bacteria and their mammalian host [83, 84]. Additionally, other researchers stated that indole, being an intercellular signaling molecule, controls numerous phases of bacterial physiology, entailing resistance to drugs, spore formation, plasmid stability, biofilm formation, and virulence [77, 80–82, 85–87]. Indole is, therefore, a bacterial signaling molecule [82].

In recent times, indole was found to inhibit E. coli cell division as a measure of a cell cycle checkpoint initiated by the build-up of plasmid dimers [82, 86–88]. Indole is also a natural proton ionophore because of its major activity to inhibition of division in the biological process [82]. Plasmid dimers yield a controlling ribonucleic acid (RNA) which instigates indole synthesis by tryptophanase enzyme [82]. Enormous numbers of Gram-positive and Gram-negative bacteria species, including E. coli, manufacture indoles as interspecies and interkingdom signaling molecules [76]. Indoles play significant actions in several bacterial phenotypes and eukaryotic immunities [76]. Specifically, indole has been reported to modify biofilm formation and persister formation in E. coli [76, 85].

On a similar note, it is noteworthy that functional groups on indole moiety control biofilm formation and have antipersister activities than indole on its own [76]. Indole derivatives play significant cellular roles, entailing neurotransmitters, such as serotonin [63, 67].

Monte et al. studied and evaluated the antibacterial activities of four phytochemicals, namely, hydroxycoumarin (7-HC), indole-3-carbinol (13C), salicylic acid (SA), and saponin (SP) against Escherichia coli and Staphylococcus aureus, either as planktonic cells or as biofilms [32]. Additionally, the four phytochemicals were used as combination therapy with three antibiotics to evaluate any synergistic impact [32]. They observed that among the four phytochemicals, 7-HC and 13C were the most active phytochemicals against E. coli and S. aureus. Both 7-HC and 13C performed significant functions in the intervention of cell-cell communications and biofilm formation and control, because they influenced the motility and quorum-sensing activities [32]. Conversely, none of the four phytochemicals eliminated the biofilm completely. This resulted to dual combinations between ciprofloxacin (CIP), erythromycin (ERY), tetracycline (TET), and 13C, which produced synergistic activities against S. aureus-resistant strains [32].

The relationship of 7-HC ERY was antagonist against bacterial strains of S. aureus CECT 976 and S. aureus RN 4220. Additionally, the dual combination of SP-TET or SP CIP offered antagonistic in different effects against S. aureus CECT 976. The 7-HC-TET against S. aureus XU 212 and SP-ERY against S. aureus CECT 976 gave synergistic (additive) effects [32]. A dual combination of 13C with all the antibiotics displayed synergistic effects against the four assessed S. aureus strains (S. aureus CECT 976 ERY, S. aureus XU 212, S. aureus RN 4220, and S. aureus SA11993). The synergistic effects were also confirmed with a dual combination of SA or SP with TET, ERY, and CIP against S. aureus XU 212, S. aureus RN 4220, and S. aureus SA11993. This fortified the merits of antibacterial activities of photochemical-antibiotic combinations [32]. In summary, the four phytochemicals possessed the potentials to regulate the growth of E. coli and S. aureus in both planktonic and biofilm statuses. Additionally, the phytochemicals confirmed their potentials to perform synergistically with old antibiotics, thereby contributing to contributing to its recycling, which was previously considered inefficient because of resistance.

Similarly, Lee et al. studied thirty-six different indole derivatives with the aim of ascertaining new compounds which could prevent bacterial persister and biofilm formation by Gram-negative E. coli and Gram-positive S. aureus [76]. Four halogenated indoles (5-iodoindole, 4-fluoroindole, 7-chloroindole, and 7-bromoindole) eliminated persister formation by E. coli and S. aureus. Among these halogenated indoles, 5-iodoindole was confirmed to be most potent to prevent biofilm formation by the two bacterial strains [76]. The reason being that 5-iodoindole did not induce persister cell formation, like the other three halogenated indoles, but prevented the manufacture of the immune-evasive carotenoid staphyloxanthin in S. aureus. As a result, 5-iodoindole reduced the manufacture of virulence factors in the strain [76]. Lee et al. concluded from their studies that halogenated indole is potentially valuable to control bacterial antibiotic resistance [76].

Based on halogens' reactivity in the periodic table, reactivity increases up the group and decreases down the group (fluorine, chlorine, bromine, iodine, and astatine): fluorine, being the first member of the halogen group (family), chlorine the second member, bromine, the third member, iodine the fourth member, and astatine the fifth member. In other words, reactivity decreases down the group because electronegativity decreases the group. Nevertheless, Lee et al.'s results are independent of the reactivity order of the halogens in the periodic table because of oxidative character, but dependent on nucleophilicity which is more likely to influence binding to active sites as an opposite trend [76]. Additionally, Lee et al. indicated that 5-iodoindole could be used in combination with commercial antibiotics to eliminate persister cells and biofilms [76].

Kemp et al. confirmed the current investigation on the signaling molecule indole as a target for quorum-sensing inhibition (QSI) and the application of indole derivative called indole-3-carboxaldehyde (ICA) as quorum-sensing inhibitor (QSI) to mediated behaviors in Escherichia coli [35]. From Kemp et al.'s study, they explored bromination as an approach to increasing the QSI of indole carboxaldehydes (ICA) abilities. The inhibition concentration at fifty percent (IC50) of 5-bromoindole-3-carboxaldehyde, 6-bromoindole-3-carboxaldehyde, and 7-bromoindole-3-carboxaldehyde was determined and compared to the IC50 value of ICA. Their results showed that the bromination of these indole carboxaldehydes reduced the IC50 values between 2- and 13-fold, which implied that bromination essentially enhanced the efficacy of all the indole carboxaldehydes [35].

## 6. Conclusion and Future Research

Biofilms are responsible for enhancing the multidrug resistance of antibacterial drugs. This paper gives a review on contextual biofilm formation, quorum sensing as a bacterial communication signal, and antibiofilm agents (quorum quenching) as eradication approaches, Phytochemicals in plants help to control and prevent biofilms. The use of indole derivatives from plants sources (phytochemicals) is the best nontoxic green chemistry approach to eliminating biofilm. Most researchers indicated combination therapy as the best approach to prevent biofilms. From these researchers' schools of thought, future research will entail a combination therapy of 5-iodoindole and eight different antibiotics to confirm synergistic results. Results will be compared with three phytochemicals found usually in cruciferous vegetables, namely, indole, indole-3-carbinol, and 3, 3′-diindolylmethane.

## Data Availability

The data in the document and figures used to support the findings on this study are included within the research article.
